RETRACTED

# Analysis of Hepatic Artery Infusion (HAI) Chemotherapy Using Randomized Trials of Floxuridine (FUDR) for Colon Cancer Patients with Multiple Liver Metastases

**DOI:** 10.1155/2022/3546455

**Published:** 2022-04-27

**Authors:** Yuanming Li

**Affiliations:** Minimally Invasive Tumor Therapies Center, Beijing Hospital, National Center of Gerontology; Institute of Geriatric Medicine, Chinese Academy of Medical Sciences, China

## Abstract

Colorectal cancer (CRC) is one of the leading causes of cancer-related death, with most of the people who have the disease developing numerous liver metastases. Sixty percent of colon cancer patients have liver metastases. Only 25% of those with resectable hepatic metastases are alive, and recurrence occurs in nearly half of these cases. Regardless of the fact that left-sided cancer has a higher rate of liver metastases, past study reveals that left- and right-sided liver metastatic colon cancer patients have different survival rates. Hepatic artery infusion (HAI) combined with systemic chemotherapy is a treatment option for patients with unresectable liver-only or liver-dominant colon liver metastases. Although HAI has only been performed in a few locations previously, this study used randomized trials of floxuridine (FUDR) to characterize patient selection and first perioperative results during the deployment of a new HAI program. In this research, we also looked at the technical aspects of placing implantable pumps and catheters for HAI chemotherapy, as well as the efficacy, morbidity, and outcomes of this therapy in colon cancer patients with numerous liver metastases. The parameters like toxicity, overall survival rate, response rate, and progression-free response for the suggested therapy are also analyzed. These findings have important implications for colon cancer adjuvant HAI chemotherapy.

## 1. Introduction

Every year, new cases of CRC identified around the world were greater than 1,000,000. CRC is the world's 3rd most frequent malignancies and the 4th leading cause of tumor death. Despite significant breakthroughs in detection, surgery, and treatment, CRC is the 2nd largest etiology of cancer mortality in the USA and other developed countries.

From Figure 1, it is observed that the people in the age group of 50-59 are largely affected by CRC when compared to the people in the age group of 30-49. People below the age of 30 are rarely affected by CRC.

Only around 20% of CRC cases have a genetic component, and some are associated to well-defined diseases like familial adenomatous polyposis and hereditary nonpolyposis CRC. Environmental variables, rather than heritable genetic changes, have been linked to the majority of CRC cases. Mutagens from the environment and food, specific gut commensals and infections, and chronic intestinal inflammation, all of which occur prior to tumor development, are all risk factors [1].

RETRACTED

CRC risk factors are classed as modifiable or nonmodifiable (family history, age, family history, inherited propensity, adenomatous polyp, and gastrointestinal illness that are both treatable and preventable). Other food-related risk parameters are smoking, diets, high alcohol consumption, and obesity. Lymphocytic and hematogenous progress, as well as contiguous and transperitoneal distribution, are all possible ways for CRCs to spread. Liver, regional lymph nodes, bones, and lung are the most common metastatic locations. A fraction of initially unresectable colorectal liver metastases (CLMs) can now be focuses to ablation or resection due to recent breakthroughs in chemotherapeutic, surgical, and interventional procedures. As a result, determining the resectability requires a precise assessment of the disease's breadth. CLM is detected using a variety of imaging methods. Computed tomography (CT), ultrasound, 18F-FDG PET/CT, magnetic resonance imaging (MRI), and integrated 18F-FDG PET/MR are all common imaging modalities.

The bulk of cancer-related deaths are caused by metastasis, which remains a therapeutic problem. Metastatic cancer cells are similar to initial cancer cells in most ways, although they may be altered by the environment of the organs they inhabit. Because of portal venous outflow from the colon, the liver is the most likely visceral metastatic location. About 15% of individuals have synchronous metastases in the liver at the assessment time, which is an unfavorable prognostic risk. When colorectal cancer cells spread and invade the liver, a critical metabolic organ, they undergo metabolic reprogramming. CRC proceeds through an adenoma-to-carcinoma sequence that finally leads to liver metastases in 60% to70% of individuals. At this point, CLM is the important cause of deaths in CRC patients, as the disease becomes more difficult to treat and finally develops resistance to most types of combination therapy [2].

Significant improvements in the CLM treatment over the last 50 years, including extremely sophisticated combinations of surgery and systemic therapy, along with earlier identification, have contributed to doubling of median survival from 25% to 50%. In the case of metastatic disease, the prognosis is improving, and around 30% of patients who have liver resection will live a long time. Most of the cancer individuals will, unfortunately, have illness recurrence. Recent studies have found a 7% enhancement in progression-free survival when systemic chemo-treatment (SC) is integrated with surgical resection for CLM. Hence, chemotherapy is now considered typical treatment [3].

RETRACTED

Several prospective randomized and nonrandomized trials have looked at the employment of regional chemo-treatment alone or in collaboration with SC to treat suspected lesions in the residual or unresected liver, which prevent the recurrence of metastases and improve survival. HAI of antimalignant medicines is one localized treatment that considers the advantage of particular properties of hepatic cancers. It is known that tumors in hepatic region obtain most of their blood through the hepatic artery (HA). On the other hand, the portal vein supplies most of the blood to normal liver cells. Because of these unique properties, a higher concentration of anticancer drugs can reach the tumor through HA and preserve the normal parenchyma of the liver. Larger local medication concentrations can be attained, while systemic effects are avoided since the liver can metabolize a wide spectrum of medicines [4].

A continuous chemotherapeutic agent infusion also increases the exposure of drug to tumorous cells, potentially raising the fraction of killing tumor cells. These ideas suggest that HAI therapies could be beneficial in the CLM treatment. A number of different chemotherapeutic drugs have been explored, both alone and in combination. Due to the attributes namely higher solubility and capability to be concentrated in a smaller volume, floxuridine (5-fluoro-2′-deoxyuridine), FUDR, is the most commonly employed agent for HAI with the implanted pump (5-fluorouracil) [5].

In our study, we analyzed the effect of HA infusion (HAI) chemotherapy using randomized trials of floxuridine (FUDR) for the treatment of CLM patients. The further organizations of the research paper are shown below.  Section 2 shows the problem statement.  Section 3 provides the methods and materials for our study. Performance evaluation is given in Section 4. The paper conclusion is given in Section 5.

## 2. Problem Statement

CRC is the 3rd most prevalent category of malignancies in the world. Approximately 60-70% patients would develop colorectal liver metastases (CLM), which are a major cause of death in greater than 50% of CLM patients. In individuals with synchronous liver metastases, the history of the disease without treatment is progression of disease with an average survival of roughly 4.5 months. Although surgical excision of these liver metastases is still the gold standard of therapy, the majority of patients have unresectable lesions. To treat the unresectable lesions, chemotherapy is the significant metastatic colorectal cancer treatment, resulting in a higher CLM survival rate. If chemotherapy drugs are injected into the HA, they can be administered directly to cancer cells which improve the effectiveness of therapy [6, 7]. Hence, HAI is a potential chemotherapy technique. FUDR is the most utilized chemotherapeutic drug due to its higher hepatic extraction rate. So, HAI-FUDR chemotherapy has a potential application in treating CLM [8].

RETRACTED

The side effects of floxuridine are chest pain or pressure, difficulty swallowing, gum, inflammation or bleeding, mouth ulcers, flu-like sensations, scratchy throat, painful mouth, and dizziness, and severe diarrhea or vomiting and coughing up the blood or vomiting that resembles coffee grounds are some of the symptoms, the appearance of purple or red patches beneath your skin, as well as easy bruising, an uncontrollable source of bleeding. We found floxuridine drug because it has more advantages then, when compared to other drugs.

## 3. Materials and Methods

Chemotherapy is a common metastatic colorectal cancer treatment for unresectable tumors, resulting in a greater CLM survival rate. Chemotherapy medications can be delivered directly to cancer cells when injected into the HA, increasing the efficiency of treatment. As a result, HAI could be used as a form of chemotherapy. The chemotherapy medication FUDR is the most widely used. This study focuses on the analysis of the effect of HAI chemotherapy using randomized trials of floxuridine (FUDR) for CLM.  Figure 2 shows the detailed flow of the work.

### 3.1. Patient Selection

The dataset for this study considers 220 patients recruited from secondary care settings in 39 Chinese National Health Service hospitals. The patients required for further study were selected from this list based on certain criteria. They should be greater than 18 years old, with WHO performance grade of 2 or less, and have CLM that was resectable or suboptimally resectable with no extrahepatic metastatic disease. The number of metastases found in CLM is not a problem. Before entering the experiment, the initial cancer had to be excised or declared resectable, according to the protocol.

Patients were not permitted to participate in the study if they possess uncontrolled health conditions that would make treatment or response assessment difficult. The following clinical parameters must be considered in selecting eligible participant.

Inclusion criteria are the following:

- Platelet count > 100 × 10^9^ per L
- Neutrophil count > 1 · 5 × 10^9^ cells per L
- Serum bilirubin < upper limit of bilirubin
- Alkaline phosphatase < upper limit of normal level
- Serum aminotransferase (alanine aminotransferase or aspartate aminotransferase) < upper limit
- Rate of glomerular filtration > 50 mL/min
- Creatinine clearance > 50 mL/min

Exclusion criteria are the following:

- No psychiatric or neurological disorder affecting ability to consent or comply with medication
- No partial or complete obstruction in the bowel
- No preexisting peripheral neuropathy of grade 1 or worse according to common toxicity criteria
- No family history of deficiency in dihydropyrimidine dehydrogenase
- Gilbert's syndrome or other abnormalities in biliary transportation should not be present

RETRACTED

### 3.2. Triphasic Computed Tomography

The triple-phase liver CT procedure can be used to diagnose localized liver lesions, hypervascular liver metastases, and endocrine malignancies. It is the most prevalent imaging modality for intrahepatic and extrahepatic lesions and also postoperative studies. CT scans, on the other hand, are insufficiently sensitive to detect lesions lesser than 1 cm in diameter. Standard triphasic CT includes three phases, namely, delayed phase, arterial phase, and portal venal phase. Average volume of Bolus injections used for this scan was 100-370 mL for a single patient, and the mean concentration of iodinated contrasting agent used was about 300-350 mg/mL. The eligible patients selected were subjected to triphase CT. The resultant CT scans of the patients were analyzed by radiologists and surgeons for detecting the presence of extrahepatic disease [9, 10]. The standard deviation of bolus injection is an epidural saline injection of 20 to 30 mL, followed by further injections if needed, and has been shown to be an effective treatment for master of public health (MPH); however, the method is hampered by an excessively high recurrence rate.

### 3.3. Preoperative Evaluation of Patients

Before starting the HAI treatment, the critically eligible patients must be chosen from the generally selected patient list obtained from the previous step, depending on specific attributes. CT scans of patients were used for the preoperative assessment of participants. The criteria for this assessment using CT scan are given as follows. Hepatic metastases must be verified histologically. The hepatic lesions must be greater than 2 cm in diameter and available as unresectable. The presence of extended liver metastases (40% replacement in hepatic region) is reported to augment 30-day laparotomy fatality from 2% to 20%, offsetting the advantages of HAI. Hence, patients must be free of extrahepatic disorders. This is evaluated by CT scans. Hepatic involvement by the CRC must be less than 75%.

Obviously, the coagulopathy and infections must be absent in participants prior to the implantation of any foreign substance. Evidence of insufficiency in liver and lesser patient performance should also be considered when making a decision. Patients who are suited for pump installation in HAI treatment can be identified using these parameters [11–13].

RETRACTED

### 3.4. HAI Chemotherapy

The goal of HAI is to make lesions exposed to high amount of antitumor agents with limiting the systemic damage. This is accomplished by injecting a medication into the HA, which mostly provides blood to tumors in hepatic sites, rather than the portal veins, which primarily provides blood to normal liver cells. The chemotherapeutic agent FUDR has been explored the most. When regularly administered in the HA, FUDR had a 95% hepatic extraction rate, leading to an increased concentration in CLM compared to SC. Hence FUDR is used as a potential chemical agent in HAI therapy of colon metastases [14].

The anticancer agent FUDR is administered into the HA with the utilization of an implantable pump for subcutaneous infusion and a surgically implanted HA catheter, which distributes the anticancer agent at a slow fixed rate for two weeks. This administration style is superior to existing conventional approaches in terms of survival rate and progression-free survival. Displacement of catheter, infections, thrombosis in HA, hematomas, and perfusion in liver are only a few of the issues associated with pumps. The technical issues are related to the surgeon's experience as well as the artery structure [15].

#### 3.4.1. Implantable Pump

Longer infusions using external pump systems are related to a number of problems. Dislodgement and sepsis of catheters, failures in the external pump, and fluctuations in the flow rate were all reported as complications. Patients' acceptance of an external catheter device that restricted their lifestyle and activities was also an important concern in addition to these issues. With the invention of the implanted pump, these issues were resolved.  Figure 3 shows the general structure of the implantable pump used in HAI.

A tubular titanium cylinder with two compartments divided by a metal bellows makes up the pump. One of the compartments is a permanently sealed fluid chamber used for charging. The chamber containing the drug is on the opposite side of the bellows, accessible through a resealable valve for drug loading. It also features a catheter-connected exit. The fluid container applied for charging consists of fluorocarbon liquid which is warmed by using the temperature of patient's body and changed to a gas phase, which keeps the drug chamber at a constant pressure [16, 17]. The pressure applied by the vapor in homeostasis with the steady liquid phase and independent of volume at a given temperature. The steady pressure forces the process of draining the anticancer agents from the chamber into the catheter with maintaining the flow rate as constant [18].

RETRACTED

When the drug in the chamber is utilized completely, percutaneous refilling compresses the gas phase stored in the charging chamber. Over external pump systems, the benefits of a drug chamber with refilling capacities, liberation from an external power supply, and a steady flow rate are considerable. Percutaneous administration through a self-sealing valve refills the inner drug chamber. The gas is compressed back to a liquid condition, allowing the pumping motion to continue. Depending on the manufacturer, the pumps can carry anywhere from 30 to 50 mL of chemotherapeutic drug and distribute at a set rate. If an aqueous solution is utilized, the manufacturer calibrates the infusion rate so that the reservoir is replenished every two weeks. The rate can be tweaked even more by adjusting the viscosity of the infused solution. The pumps are also engineered to provide you easy accessibility to the catheter while or after it has been placed, so you can flush it or undertake angiographic investigations [19].

#### 3.4.2. Catheters

Port-catheters can be placed through surgery. The catheter is inserted during a laparotomy, which is commonly performed after the primary tumor is removed. This methodology enables for surgical investigation of the entire abdomen, prophylactic artery ligature to prevent prophylactic cholecystectomy (to avoid chemical cholecystitis), extrahepatic infusions, and quality control of perioperative infusion with blue or fluorescein injections through the catheter [20]. The radiological techniques employ percutaneous radiologic insertion into the femoral artery. The tip of the catheter is inserted and embolized in the gastroduodenal artery (GDA). To facilitate the infusion into the HA, the catheter is pierced on one side, and a side hole is placed. The catheter is linked to a subcutaneous portal after a control arteriography for easy access and repeat infusions. There is no significant difference in effectiveness or local complications associated between surgical and radiologic implantation, according to retrospective analyses. It is, however, becoming increasingly common due to its ease of use and a trend toward extended life of catheters and a lesser risk of complications after the radiologic implantation. A catheter implantation staff with a lot of experience is necessary [21].

#### 3.4.3. Placement of Catheters and Pumps

Catheter placement requires a dilated transverse arteriotomy to prevent the development of an intimal flap during the insertion of catheter into ligated GDA. The catheter is tied to a bead which is placed closer to the catheter tip with a ligature. The catheter will not fall into the common HA (CHA) or out of the GDA if this is done. The tip of the catheter should be placed where GDA exits CHA. A vascular clamp applied during the catheter's entrance into GDA will ensure the presence of catheter's tip in GDA [22]. Another important step in avoiding misperfusion in duodenum and stomach is GDA devascularization, which involves ligating vascular tissues along the superior walls of the duodenum and stomach starting from the lower portion of stomach to the bile duct. The liver's collateral blood flow allows for the blockage of abnormal lobar arteries and the following crossover perfusion by vessels which are nonligated. In the case of abnormal HA architecture, this makes catheter placement easier [23].

RETRACTED

A pump pocket is formed in any of the lower abdomen portion. The catheter is routed to connect the pump pocket that is formed newly through the shortest peritoneal break possible to prevent leakage in ascites. This must be done before the catheter is inserted into HA [24]. The pump is attached to the pocket's floor by sutures placed in the abdominal wall. If the participant is highly obese, insertion of the pump pocket in the lower belly wall will make the accessing process to encounter the pump harder due to the presence of thick pannus. Positioning the pump pocket above the area of lateral rib cage is another option. The pump was placed in a subcutaneous pouch in the right lower abdominal quadrant. Fluorescein dye was introduced into the side port of pump to determine the amount of dye taken up by the liver and to rule out extrahepatic perfusion.

#### 3.4.4. Randomized Clinical Trials Using FUDR

The chemotherapeutic agent FUDR has gotten the greatest attention. FUDR exhibited a 95% of liver extraction rate when injected regularly in the HA, which results in a greater concentration in CLM compared to SC. As a result, FUDR is being investigated as a possible chemical agent for HIA therapy of colon metastases. In comparison to other agents, FUDR is the most extensively employed agent for HAI with the embedded pump due to its solubility qualities and capacity to be concentrated in a lesser volume [14].

Patients were randomly assigned to either of two categories, namely, the testing group and the control group. The testing group has 122 samples, and the control group has 98 samples. The initial FUDR dose was 0.3 mg/kg/d for a 14-day course, followed by two weeks of regular normal saline administration. When the pump reservoir of 50 mL capacity was supplied with the medication or saline, 10,000 U of heparin was added. Patients in the testing group receive FUDR through the hepatic arteries [25].

RETRACTED

#### 3.4.5. Systemic Chemotherapy

Anticancer medications are injected into the vein during systemic chemotherapy (SC) [26]. These medications go throughout the body by means of blood flow. SC was administered to the control group. The control group (no HAI) received a 14-day cycle of systemic injection of FUDR at 0.3 mg/kg/d through portal veins, followed by two weeks of regular normal saline administration [3].

## 4. Results and Discussion

The effect of HAI using FUDR on the treatment of CRC patients with multiple liver metastases was studied and compared to that of systemic chemotherapy using FUDR in terms of survival rate and progression-free survival rate. The testing group and control group were subjected to HAI-FUDR and systemic FUDR therapies, respectively.

The overall survival rate (OSR) of HAI-FUDR and systemic FUDR treatments was compared in Figure 4. OSR is defined as the proportion of people in a treatment group who are still surviving after being diagnosed with cancer or commencing treatment for it after a certain amount of time has passed (generally five years). It is evident from Figure 4 that OSR was significantly improved when a patient was treated with HAI-FUDR therapy when compared to that of patient treated with systemic FUDR therapy. This tells that number of participants who survive after five years of chemotherapy is increased in case of HAI-FUDR therapy compared to that in systemic FUDR cases. Hence, quality of patient's life is better when HAI-FUDR is used as treatment option for colorectal liver metastases.  Table 1 shows the toxicities exhibited in patients during HAI-FUDR and systemic FUDR treatments. Number of patients affected with described toxicities was lesser in case of HAI-FUDR treatment compared to that in systemic FUDR therapy.

Figure 5 shows the graphical analysis of overall progression-free survival (PFS) rate in HAI-FUDR and systemic FUDR approaches. PFS is defined as the period a patient survives with cancer, during and after therapy, during which the disease does not worsen. PFS rate is a significant indicator of effectiveness of a treatment. It is clear from the Figure 5 that overall PFS rate is improved in case of HAI-FUDR when compared with that of systemic FUDR. Improved overall PFS rate indicates that worsening of colorectal and liver regions in HAI-FUDR-treated patients is significantly lesser. In addition, this indicates that the formation of new lesions, further dispersal of tumor, and growth speed of tumor are significantly lesser in HAI-FUDR-treated patients.  Figure 6 shows the graphical analysis of hepatic progression-free survival rate in HAI-FUDR and systemic FUDR approaches. It is clear from Figure 6 that hepatic PFS rate is improved in case of HAI-FUDR when compared with that of systemic FUDR. Improved hepatic PFS rate indicates that worsening of liver regions in HAI-FUDR-treated patients is significantly lesser.

RETRACTED

Table 2 shows the overall response rate (ORR) attained in HAI-FUDR and systemic FUDR therapies. ORR is defined as the percentage of individuals whose tumors reduce in size (partial recovery) or disappear (completely recovered) after treatment. High response rate is observed in HAI-FUDR cases compared to that in systemic FUDR cases. This tells that HAI-FUDR therapy can efficiently treat the hepatic lesions.

## 5. Conclusion

CRC remains the 3rd most typical tumor in the world with greater than half of the cases possess liver metastasis. Most of the patients with CLM experience recurrence after resection of tumor segments. The utilization of chemotherapy after resection for CLM has a significant advantage. The capacity to provide higher concentrations of chemotherapeutic component continuously by means of HA compared to systemic chemotherapy paved way for the potential application of HAI in treating CLM. In this paper, we studied the effect of HAI therapy using FUDR as chemotherapeutic agent in CLM patients. The employment of HAI chemotherapy using FUDR has been shown to extend the normal quality of life compared to systemic chemotherapy. This conclusion is made from the analysis of parameters, namely, OSR, PFS rate, and ORR. Because of the emergence of the implanted pump, the therapy is now mechanically viable and agreeable to patients. Hence, it is evident that the utilization of HAI-FUDR has a potential application in the recovery of patients with CLM compared to systemic chemotherapy. In the future, multiple trials of HAI-FUDR chemotherapy (combination of FUDR with other chemotherapeutic agents) must be carried out to enhance and study the efficiency and safety of HAI-FUDR chemotherapy. Research must be done to reduce the level of toxicities resulted in HAI-FUDR therapy.

## Figures and Tables

**Figure 1:** Prevalence of CRC.

**Figure 2:** Detailed flow of the proposed study.

**Figure 3:** Structure of implantable pump.

**Figure 4:** Overall survival comparing HAI and systemic chemotherapy.

**Figure 5:** Comparison of overall progression-free survival rate.

**Figure 6:** Analysis of Hepatic progression-free survival rate.

**Table 1:** Treatment toxicities.

Variables	Number of patients affected (%)	
	Systemic FUDR	HAI-FUDR
*Chemotherapy related*		
Vomiting	65%	50%
Diarrheal	46%	35%
Mucositis	36%	20%
Rash	24%	20%
Neurotoxicity	63%	55%
Thrombocytopenia	59%	45%
Anemia	44%	35%
Neurotoxicity	82%	78%
High blood pressure	6%	5%
*HAI/catheter-related*		
Pain during HAI	46%	43%
Extrahepatic perfusion	28%	25%
Catheter dysfunction	47%	35%

RETRACTED

**Table 2:** Overall response rate observed in chemotherapy approaches.

Chemotherapy approaches	Response rate (%)
HAI-FUDR	60%
Systemic FUDR	45%

## Data Availability

The analyzed datasets generated during the study are available from the corresponding author upon request.
